# The Practices of Solid Waste Utility and Thriving Conditions of Logistics (a Case of Tepi Town): A Study to Treat the Healthy Environment

**DOI:** 10.1155/2022/8391616

**Published:** 2022-07-09

**Authors:** Ngiste Amare, Ola Al-Bhadly, Mequanint Birhan, Sana Sulaiman Hamid, A. Abdullah. H. Mohamad

**Affiliations:** ^1^Department of Civil Engineering, Mizan Tepi University, Tepi, Ethiopia; ^2^Department Medical Laboratory Technique, Dijlah University College, Baghdad, Iraq; ^3^Department of Mechanical Engineering, Mizan Tepi University, Tepi, Ethiopia; ^4^Al-Farahidi University, Communication Technical Engineering, Baghdad, Iraq; ^5^The University of Mashreq, Research Center, Baghdad, Iraq; ^6^Department of Medical Laboratory Techniques, Al-Turath University College, Baghdad 10021, Iraq

## Abstract

Unwanted remains, discarded residues, and byproduct materials that are not required by the initial user are known as wastes. In Ethiopia, improper solid waste management becomes endemic and it affects the health conditions, comforts, and freedom of town communities. Improper solid waste management can also adversely affect infrastructure damages, socioeconomic conditions, and environmental and health problems. So, awareness creation among the communities is necessary. The main objective of the study was to assess the management of existing solid waste activities and reverse logistic systems in Tepi town. The impacts of improper solid waste management were reduced through waste accumulation, transportation, recycling, and waste removal. Available pieces of information for the study were gathered from 450 near house places and 549 survivals. The collected data were analyzed by using Vensim system dynamics software, and the obtained results were modeled by a system dynamic cause and effect relationship diagram. Finally, the appropriate recommendations for communities, municipals, and institutions were provided.

## 1. Introduction

Unwanted remains, discarded residues, and by-products of materials that are not required by the initial users are called wastes [1]. Governments are investing huge amounts of money and many countries are battling with waste management to tackle waste issues all over the world [2]. The rapid urbanization and population growth have a great effect on the municipal solid waste generation rate [3]. Independent and intensive explorations and research on municipal solid waste collections were conducted by developed countries, and they can reach an effective waste collection process with a performance rate of 100% [4]. Countries like China, Singapore, the Netherlands, and Sweden can also reduce waste through the concept of reuse and recycling with a performance rate of 25% [5]. Landfilling and burning management of solid wastes in Israel and Slovakia affect environmental health [6]. In urban centers, about 95% of the collected solid wastes were thrown away at dumping sites and less than 50% were collected [7].

In cities and towns of developing countries, solid waste management deficiencies were visible in many areas with little or no attention in those urban centers at all [8]. 30–50% of the generated urban center solid wastes of developing cities were thrown away on streets and open spaces causing serious health problems [9]. This is due to the lack of sufficient solid waste collection services [10]. In low-income countries, more than 50% of the collected solid wastes were disposed of on uncontrolled landfilling and the collection rates reached about 70% [11]. Due to the concentration of industries, an urban population growth, the consumption of residents, and inadequate finance and facilities, the volume of waste was increased in urban areas of SNNPR [12]. In Tepi town, the generated solid wastes were thrown away on streets, unapproved dumpsites, in waterways (drainage systems), and at open sites near the residential areas affecting the environment [13].

Solid wastes that are carelessly disposed of and end up everywhere can poison and contaminate the world [14]. So, these contaminations can cause water, soil, and air pollution which leads to global warming [15]. The polluted water chemicals will damage plants and fish in lakes. Inadequately managed landfills may cause air and other environmental pollution across the world [16]. The health, well-being of residents in cities and towns of urban areas, and the environmental protections were kept by adequate solid waste facilities [17]. The town municipality's commitments and active involvements of the communities have a significant role in managing the solid wastes properly [18]. This study assessed the Tepi town's solid waste management adoption practices. If solid waste is not effectively managed, it hurts the environment and public health [19]. Otherwise, if it is managed properly, it can be a valuable resource [20]. This study assessed the contributing factors, the impacts, the role of the logistics process, and the improper management activities of the solid wastes in Tepi town.

The outcomes of the study help in developing solid waste management problem-solving policies for the local policymakers. It is also used for conducting a similar study at a regional level. Solid waste management improves the development and progress of any country [21]. However, this study shows that both the services and the practices of managing solid waste were poor at the household and municipality levels. Hence, solid waste management plans and strategies should be developed by the municipality of the town to improve the services, public awareness, public participation, and public involvement and to enforce the laws and regulations.

## 2. Objective

### 2.1. General Objective

The objective of the study is to search the solid waste management practices of Tepi town in three kebeles, reverse logistics of wastes, and waste disposals to reduce improper management of solid wastes and their impacts on health and the environment.

### 2.2. Specific Objectives

The specific objectives are as follows:

- To assess the existing practices of the solid waste management
- To identify influencing factors for the improper management of the solid wastes
- To investigate an improper solid waste management impact
- To be aware of the role of logistics in the management activities of the solid wastes

## 3. Methodology

### 3.1. Study Area

Tepi is among the Ethiopian towns found in the southwest of Ethiopia at 621 km south of Addis Ababa on a latitude of 7°12′N, a longitude of 35°27, and an elevation of 1097 meters above mean sea level [22]. The town is well known for coffee and spice production [23]. Tepi town has three known kebeles: Hebert, Andenet, and Selam kebeles.

### 3.2. The Type of Research

Due to the nature of the study, mixed type of research was employed.

### 3.3. Data Sources and Data Collection

Primary data: from direct observation, existing dried and semiliquid dirt will be captured through the camera. An in-depth interview and the designed questionnaire were distributed to key informant respondents. The secondary data sources were referred to and collected from books, journals, and other unpublished research studies.

### 3.4. Sampling Size and Technique

The sample size determination formula is taken from the Cochran formula [24].

*N* = (*Z*^2^(*pq*))/*e*^2^, where *N* is the total number of directly effaceable population size, the margin error (*e*) is 0.03, the confidence level (*Z*) is 99%, and the target design will satisfy 85%. Stratified sampling targets will implement according to key informant groups.

### 3.5. Data Analysis and Presentation

System dynamics, Excel, and Microsoft word were used. Tables, graphs, and logical arguments by narration were utilized. From captured data in the community, the researcher recorded directly in Tepi town all kebeles as a sample. It is shown in Figure 1 for clarification.

## 4. Results and Discussion

The survey study design was conducted in the near house places of Tepi town. The required data were collected from 450 near house places and 549 respondent individuals of the three kebeles through a multistage sampling technique. Then, the collected data were analyzed by SPSS statistical analysis software. Bivariate and multivariate analyses were done to identification of the good practices of solid waste management predictors. The level of significance between determinant factors was assessed by using the odds ratio with a 90% confidence interval and *p* value < 0.05. A 92% response rate was achieved; 366 out of the 549 questionnaires sent out were returned. Descriptive statistics were used for reporting the analyzed results.

The outcomes of the study show that the management practices of solid waste in the majority of the households were poor. The age of the respondents was significantly correlated with the management practices of the household solid wastes in the study area. A second analysis was done by Vensim (system dynamics software), and the factors considered are community attitude, municipal commitment, intellectual contribution, phenomena, and lack of infrastructure in the town. The basic cause-effect relationship analysis was done using the following five factors. Those are solid waste quantity in Tepi town, dirt accumulation, dirt removal, waste management practices, reverse logistic system, kinds of businesses, and then finally wastage rate.

From Figure 2, it is possible to grasp the causes and root causes that affect the rate of the waste. Due to that, there is an impact on health and environmental pollution problems. The result implies that it is better to check and control the root causes rather than focusing on the effects. The study contributes to knowledge of the subjects of solid waste management outcomes. For data analysis and interpretation, the computations of the standard deviations and the means, together with the structural equation model, have also been used. From this study, the solid waste management practices were associated with homeownership, attitude, education level, and cleanup campaign participation. Therefore, continuous awareness creation companies and community-based programs were needed to increase the coverage of door-to-door collection services of the solid wastes and encourage the ability of recycling and proper solid waste disposal by the households.

## 5. Conclusion and Recommendation

In this study, the data were gathered from only one town (Tepi), the respondent responses may be biased, and the attitudes of the respondents may also be misinterpreted. So, those were the limitations of the study, and it is better to collect the data from different cities. In addition to this, the number of participants and the sample size were also not sufficient enough. In the future, it is better to call all stakeholders and shareholders to participate in both genders in an equal ratio better to take. In this research, no governmental support or environmental specialist was included. Since the current study was conducted during the recession-era, the results found on the suffering period may be different.

Last, it is better to use more variables than the variables that were included in this study to obtain a better result. So, it is recommended to conduct other vast and frequent longitudinal research and managerial support to Tepi town at the zonal level and woreda level.

## Figures and Tables

**Figure 1:** Different kinds of sample wastes in Tepi town.

**Figure 2:** System dynamics model of the factors.

## Data Availability

The data used to support the results of this study are included within the article.

## References

[1] Tanskanen P. (2013). Management and recycling of electronic waste. *Acta Materialia*.

[2] Berry M. A., Rondinelli D. A. (1998). Proactive corporate environmental management: a new industrial revolution. *Academy of Management Perspectives*.

[3] Achankeng E. Globalization, urbanization and municipal solid waste management in Africa.

[4] Purwani A., Hisjam M., Sutopo W. (2020). Municipal solid waste logistics management: a study on reverse logistics. *AIP Conference Proceedings*.

[5] Nnorom I. C., Osibanjo O. (2008). Overview of electronic waste (e-waste) management practices and legislations, and their poor applications in the developing countries. *Resources, Conservation and Recycling*.

[6] Karak T., Bhagat R. M., Bhattacharyya P. (2012). Municipal solid waste generation, composition, and management: the world scenario. *Critical Reviews in Environmental Science and Technology*.

[7] Alshammari G., Hamad A. A., Abdullah Z. M. (2021). Applications of deep learning on topographic images to improve the diagnosis for dynamic systems and unconstrained optimization. *Wireless Communications and Mobile Computing*.

[8] Ogwueleka T. (2009). Municipal solid waste characteristics and management in Nigeria. *Journal of Environmental Health Science and Engineering*.

[9] Gelan E. (2021). Municipal solid waste management practices for achieving green architecture concepts in Addis Ababa, Ethiopia. *Technologies*.

[10] Lema G., Mesfun M. G., Eshete A., Abdeta G. (2019). Assessment of status of solid waste management in Asella town, Ethiopia. *BMC Public Health*.

[11] Mourshed M., Masud M. H., Rashid F., Joardder M. U. H. (2017). Towards the effective plastic waste management in Bangladesh: a review. *Environmental Science & Pollution Research*.

[12] Hasan Hameed A., Annon Mousa E., Abdullah hamad A. (2018). Upper limit superior and lower limit inferior of soft sequences. *International Journal of Engineering & Technology*.

[13] Mekonnen B., Haddis A., Zeine W. (2020). Assessment of the effect of solid waste dumpsite on surrounding soil and river water quality in Tepi town, Southwest Ethiopia. *Journal of Environmental and Public Health*.

[14] Mohiuddin A. K. (2018). Medical waste: a nobody’s responsibility after disposal. *International Journal of Environmental Sciences & Natural Resources*.

[15] Khan M. A., Ghouri A. M. (2011). Environmental pollution: its effects on life and its remedies. *Researchers World - Journal of Arts Science and Commerce*.

[16] Khadidos A., Khadidos A., Mirza O. M., Hasanin T., Enbeyle W., Hamad A. A. (2021). Evaluation of the risk of recurrence in patients with local advanced rectal tumours by different radiomic analysis approaches. *Applied Bionics and Biomechanics*.

[17] Bai X., Nath I., Capon A., Hasan N., Jaron D. (2012). Health and wellbeing in the changing urban environment: complex challenges, scientific responses, and the way forward. *Current Opinion in Environmental Sustainability*.

[18] Ahmed S. A., Ali S. M. (2006). People as partners: facilitating people’s participation in public-private partnerships for solid waste management. *Habitat International*.

[19] Ifeoluwa O. B. (2019). Harmful effects and management of indiscriminate solid waste disposal on human and its environment in Nigeria: a Review. *Global Journal of Research and Review*.

[20] Cheng H., Hu Y. (2010). Municipal solid waste (MSW) as a renewable source of energy: current and future practices in China. *Bioresource Technology*.

[21] Thi N. B. D., Kumar G., Lin C.-Y. (2015). An overview of food waste management in developing countries: current status and future perspective. *Journal of Environmental Management*.

[22] Dejene Nage G. (2018). Estimation of monthly average daily solar radiation from meteorological parameters: sunshine hours and measured temperature in Tepi, Ethiopia. *International Journal of Energy and Environmental Science*.

[23] Amamo A. A. (2014). Coffee production and marketing in Ethiopia. *European Journal of Business and Management*.

[24] Ahmad H., Halim H. (2017). Determining sample size for research activities. *Selangor Bus. Rev., *.

